# Euphorbia bicolor (*Euphorbiaceae*) Latex Phytochemicals Induce Long-Lasting Non-Opioid Peripheral Analgesia in a Rat Model of Inflammatory Pain

**DOI:** 10.3389/fphar.2019.00958

**Published:** 2019-09-03

**Authors:** Paramita Basu, Sirima A. Tongkhuya, Taylor L. Harris, Angela R. Riley, Camelia Maier, John Granger, Jennie Wojtaszek, Dayna L. Averitt

**Affiliations:** ^1^Department of Biology, Texas Woman’s University, Denton, TX, United States; ^2^American Institute of Toxicology (AIT) Laboratories, A HealthTrackRx Company, Denton, TX, United States

**Keywords:** analgesia, diterpenes, *Euphorbia*, flavonoids, hyperalgesia, inflammation, TRPV1, UPLC-ESI-MS/MS

## Abstract

The negative side effects of opioid-based narcotics underscore the search for alternative non-opioid bioactive compounds that act on the peripheral nervous system to avoid central nervous system-mediated side effects. The transient receptor potential V1 ion channel (TRPV1) is a peripheral pain generator activated and sensitized by heat, capsaicin, and a variety of endogenous ligands. TRPV1 contributes to peripheral sensitization and hyperalgesia, in part, *via* triggering the release of proinflammatory peptides, such as calcitonin gene-related peptide (CGRP), both locally and at the dorsal horn of the spinal cord. Ultrapotent exogenous TRPV1 agonists, such as resiniferatoxin identified in the latex of the exotic *Euphorbia resinifera*, trigger hyperalgesia followed by long lasting, peripheral analgesia. The present study reports on the analgesic properties of *Euphorbia bicolor*, a relative of *E. resinifera*, native to the Southern United States. The study hypothesized that *E. bicolor* latex extract induces long-lasting, non-opioid peripheral analgesia in a rat model of inflammatory pain. Both inflamed and non-inflamed adult male and female rats were injected with the methanolic extract of *E. bicolor* latex into the hindpaw and changes in pain behaviors were reassessed at various time points up to 4 weeks. Primary sensory neuron cultures also were treated with the latex extract or vehicle for 15 min followed by stimulation with the TRPV1 agonist capsaicin. Results showed that *E. bicolor* latex extract evoked significant pain behaviors in both male and female rats at 20 min post-injection and lasting around 1–2 h. At 6 h post-injection, analgesia was observed in male rats that lasted up to 4 weeks, whereas in females the onset of analgesia was delayed to 72 h post-injection. In sensory neurons, latex extract significantly reduced capsaicin-evoked CGRP release. Blocking TRPV1, but not opioid receptors, attenuated the onset of analgesia and capsaicin-induced CGRP release. Latex was analyzed by mass spectrometry and eleven candidate compounds were identified and reported here. These findings indicate that phytochemicals in the *E. bicolor* latex induce hyperalgesia followed by peripheral, non-opioid analgesia in both male and female rats, which occurs in part *via* TRPV1 and may provide novel, non-opioid peripheral analgesics that warrant further examination.

## Introduction

Scientists are in a continuous search for safe and potent analgesic drugs for the treatment of painful conditions in both men and women. Patients with intense pain is most commonly treated with a combination of systemic opioids (such as fentanyl and morphine), aspirin, and nonsteroidal anti-inflammatory drugs (NSAIDs) (Slater et al., 2010). Despite substantial advances in pain research and treatment, the negative side effects of opioids and NSAIDs remain a significant challenge to long-term pain management. Opioids cause physical dependency, tolerance, and addiction (Carter et al., 2014) while NSAIDs cause gastrointestinal disorders (Fiorucci et al., 2001). Opioid therapy also adversely affects the cardiovascular, endocrine, gastrointestinal, immune, musculoskeletal, respiratory, and central nervous systems (Baldini et al., 2012).

Pain is relayed to the spinal cord by excited nociceptors, which are the nerve endings of sensory neurons that specialize in detecting chemical, mechanical, and thermal damage to tissues. Chemicals, such as bradykinin, extracellular protons, nerve growth factor, and serotonin, are released from damaged epithelial cells and immune cells to excite nociceptors (Woolf, 1983; Julius and Basbaum, 2001; Drdla and Sandkuhler, 2008). Nociceptor excitation is then relayed to the dorsal horn of the spinal cord and ascends to the brain where the perception of pain is created. Pain behaviors can be measured as the degree of allodynia (increased sensitivity to non-noxious stimuli) and/or hyperalgesia (increased sensitivity to noxious painful stimuli). Pain therapeutics can then target the brain or the spinal cord to centrally block pain perception or the nociceptors can be directly targeted to peripherally block pain transmission.

A subpopulation of nociceptors expresses the thermosensitive transient receptor potential vanilloid 1 (TRPV1) ion channel, which can be sensitized by inflammatory mediators resulting in the amplification of pain signaling. TRPV1 is a non-selective cation channel with high permeability to calcium ions (Ca^2+^) and is expressed in the peripheral and central terminals of small diameter sensory neurons (Caterina et al., 1997; Tominaga et al., 1998; Clapham, 2003; Dinh et al., 2004; Lazzeri et al., 2004; Venkatachalam and Montell, 2007) TRPV1 is activated by heat (> 42°C), acidic pH (pH 6.0 or less) (Jordt et al., 2004) or alkaline pH (pH 7.8 or more) (Dhaka et al., 2007), and chemicals, such as capsaicin (Caterina et al., 1997), arachidonic acid metabolites (Hwang et al., 2000), N-arachidonyl dopamine (Huang et al., 2002), oxidized linoleic acid metabolites 9- and 13-hydroxyoctadecadienoic acid (9- and 13-HODE) (Patwardhan et al., 2010), and resiniferatoxin (RTX; from the latex of *Euphorbia resinifera*) (Szallasi and Blumberg, 1990; Premkumar and Ahern, 2000; Raisinghani et al., 2005). TRPV1 can also be sensitized by various inflammatory mediators (Shu and Mendell, 1999; Premkumar and Ahern, 2000; Hu et al., 2002; Sugiura et al., 2002; Sathianathan et al., 2003; Kim et al., 2004; Donnerer et al., 2005; Van Buren et al., 2005; Stein et al., 2006).

Activation and sensitization of TRPV1 leads to calcium influx and depolarization of the sensory neuron membrane followed by rapid desensitization of TRPV1, resulting in diminished action potential firing (Caterina et al., 1997) and desensitization results in analgesia. The ultrapotent TRPV1 agonists RTX causes temporary ablation of TRPV1-expressing nociceptors to produce longer-lasting analgesia (Appendino and Szallasi, 1997; Wong and Gavva, 2009; Mitchell et al., 2010; Ohbuchi et al., 2016; Salas et al., 2017). RTX was isolated from the latex extract of *E. resinifera* (*Euphorbiaceae*), which belongs to the same family with *Euphorbia bicolor*. The genus *Euphorbia* is the third largest genus of flowering plants with almost 2,000 species worldwide that are distinguishable by the presence of milky latex (Rafael Govaerts et al., 2000; Horn et al., 2012). Several *Euphorbia* species contain biologically active phytochemicals with medicinal properties (Shi et al., 2008; Vasas and Hohmann, 2014). In addition to *E. resinifera*, analgesic and/or anti-inflammatory activities have been reported in the stem extract of *E. antiquorum* (Hoang et al., 2008), hydro-alcoholic extract of *E. tirucalli* root (Palit et al., 2018), different solvent extractions of *E. dracunculoides* (Majid et al., 2015), and several other species (Prabha et al., 2008; Gaur et al., 2009; Upadhyay et al., 2014; Sdayria et al., 2018).

Snow-on-the-prairie, *E. bicolor* Engelm. & A. Gray, a relative of *E. resinifera*, is native to the Southern United States, and possesses latex similar to that found in other *Euphorbia* plants with medicinal properties. To date there are no reports on the potential medicinal properties of *E. bicolor* latex extract. Being in the same family with *E. resinifera*, which has a literature of one of its phytochemicals providing pain relief, we hypothesized that *E. bicolor* latex extract contains phytochemicals that induce long-lasting, non-opioid peripheral analgesia in a rat model of inflammatory pain. The present study is the first to report on the analgesic properties and phytochemicals of the genus *E. bicolor*.

## Materials and Methods

### Plant Collection and Extract Preparation

*Euphorbia bicolor* (*Euphorbiaceae*) plants were collected from prairies in Denton County, TX, USA. The collected plant material was identified by members of the Native Plant Society of Texas, Trinity Forks Chapter, and a voucher specimen was deposited in the TWU Herbarium. Fresh latex was collected from plucked leaves, inflorescence bracts, and cut stems in a pre-weighed vial, extracted in 80% methanol (1:40 w/v) at room temperature for two days, and centrifuged at 3,500 rpm for 20 min. Supernatants were filtered through Whatman #54 filter paper, the pH was measured at pH 5.6, and nitrogen gas was flushed into the vial to prevent oxidation before storage at −20°C for further use. After performing serial dilution of the extract, the final methanol concentration in the working solutions for *in vivo* and *in vitro* experiments was 1.2% and their pH ranged from pH 5.96 to pH 6.6.

### Animals

A total of 216 male and female adult Sprague-Dawley rats (250–350 g; Charles River Laboratories, Wilmington, MA, USA) were used in this study. The rats were separated by sex and housed in groups of two per cage in a 12:12 h light:dark cycle with *ad libitum* access to food and water. The rats were acclimated to the animal facility for a minimum of five days before conducting the experiments. All studies were conducted under the approval of the Texas Woman’s University Institutional Animal Care & Use Committee and under the strict guidelines of Animal Welfare Act, implementing Animal Welfare Regulations, and the principles of the Guide for the Care and Use of Laboratory Animals. The study also followed the guidelines of the Committee for Research and Ethical Issues of the International Association for the Study of Pain. For all behavior testing, experimenters were blind to the treatment groups during testing.

### Complete Freund’s Adjuvant

To induce hindpaw inflammation, all rats received one plantar injection of complete Freund’s adjuvant (100 μl 1:1 in 0.9% sterile saline; CFA; Sigma Aldrich, St. Louis, MO, USA) into the right hindpaw. Twenty-four hours post-CFA injection, pain behaviors (thermal hyperalgesia and mechanical allodynia, see below) were confirmed prior to further experimentation.

### Thermal Hyperalgesia

Thermal sensitivity was detected using the Plantar Test (Ugo Basile; Collegeville, PA, USA), as previously described (Hargreaves et al., 1988). For this test, rats were individually placed into non-restricting plexiglass chambers on a solid glass tabletop. A noxious heat source was aimed at the plantar surface of the rat hindpaw and the time required to elicit a paw withdraw was measured in seconds and recorded as a paw withdrawal latency (PWL). A maximum time of 20 s was allotted to prevent potential tissue damage in instances where the animal did not withdraw. Each time point is reported as an average of three trials conducted in a nonconsecutive order to prevent temporal summation of heat. Male and female rats were first acclimated to the apparatus 24 h prior to testing. Following baseline measurements (0 time point), rats received one intraplantar hindpaw injection of *E. bicolor* latex extract (25, 50, 100, 300, or 500 µg/ml in 100 µl 0.9% sterile saline and 1.2% methanol; n= 5–6 per treatment/sex) or vehicle (100 µl 0.9% sterile saline and 1.2% methanol; n= 5–6/sex). Paw withdrawal latencies were then reassessed at 20, 40, 60 min, 2 h, and 4 h post-injection.

To test whether thermal hyperalgesia is occurring *via* TRPV1, a separate set of male rats received one intraplantar injection of the TRPV1 antagonist capsazepine (10 μM in 100 µl 0.9% sterile saline and 10% DMSO; CZP; n = 7) or vehicle (100 µl 0.9% sterile saline and 10% DMSO; n = 7) into the hindpaw following baseline testing. Fifteen minutes post-injection, all rats were injected into the same hindpaw with the *E. bicolor* latex extract (300 μg/ml in 100 µl 0.9% sterile saline and 1.2% methanol) and PWL were reassessed 20 min later. The concentration and timing of CZP injections was chosen based on previous studies (Liu and Simon, 1997; Qi et al., 2015).

To test whether *E. bicolor* latex extract evoked analgesia, basal thermal sensitivity was recorded followed by one intraplantar CFA injection (see above) into the right hindpaw. Twenty-four hours later, post-CFA thermal hyperalgesia was confirmed followed by an intraplantar injection into the inflamed hindpaw of either *E. bicolor* latex extract (300 μg/ml in 100 μl 0.9% sterile saline and 1.2% methanol; n = 7 males, n = 9 females) or vehicle (100 μl 0.9% sterile saline and 1.2% methanol; n = 6 males, n = 8 females). Thermal hyperalgesia was then reassessed at 1, 3, 6, 24, 48, and 72 h post-latex injection followed by every week for 4 weeks.

To test whether analgesia was occurring *via* TRPV1, a separate group of male and female rats were pretreated with either CZP (10 μM in 100 μl 0.9% sterile saline; n = 8 males, n = 6 females), the TRPV1 antagonist 5’-Iodoresiniferatoxin (0.02 μM in 100 µl 0.9% sterile saline and 10% DMSO; I-RTX; n = 6 / sex) (Balonov et al., 2006), or vehicle injections (100 μl 0.9% sterile saline; n = 12 males, n = 12 females) into the inflamed paw (Liu and Simon, 1997; Qi et al., 2015). Fifteen minutes later, all rats received an injection of the latex extract (300 μg/ml in 100 μl 0.9% sterile saline and 1.2% methanol) into the inflamed hindpaw and thermal hyperalgesia was reassessed at 1, 3, 6, 24, 48, and/or 72 h.

To test whether analgesia occurring *via* opioid receptors, a separate group of male rats received either a subcutaneous injection of the broad-spectrum opioid antagonist naloxone hydrochloride (1 mg/kg; Sigma-Aldrich; n = 6) or vehicle (100 μl 0.9% sterile saline and 1.2% ethanol; n = 6) 24 h following CFA injections. Fifteen minutes later, all rats received an injection of either *E. bicolor* latex extract (300 μg/ml in 100 μl 0.9% sterile saline and 1.2% ethanol) or vehicle (100 μl 0.9% sterile saline and 1.2% ethanol) into the inflamed hindpaw. Thermal hyperalgesia was then reassessed by measuring PWLs at 1, 6, and 24 h post-extract injection. The naloxone dosage, injection route, and timing were chosen based on previous studies (LaPrairie and Murphy, 2007).

### Mechanical Allodynia

The Dynamic Plantar Aesthesiometer (Ugo Basile Collegeville, PA, USA) was used to measure changes in sensitivity thresholds to a non-noxious mechanical stimulus by assessing the force (in grams) required to elicit a paw withdraw from the stimulus, as previously described (Gibbs et al., 2006). For this test, rats were placed in a Plexiglas box on an elevated grid platform and a blunt probe was aimed at the plantar surface of the hindpaw. The force of the stimulus was increased with a ramp of 3 g/s over 10 s with a cutoff of 30 g to avoid mechanical lifting of the paw by the device. The average force required to elicit a paw withdrawal over 3 trials was recorded for each time point. In order to minimize the number of animals used in this study, the same animals tested for thermal hyperalgesia were also tested for mechanical allodynia. Treatment groups were counterbalanced so that each animal that received the experimental treatment in one hindpaw for testing thermal hyperalgesia, then received the vehicle treatment in the other hindpaw for testing mechanical allodynia, and *vice versa*. A period of 4 h was retained between thermal hyperalgesia testing and mechanical allodynia testing to avoid behavioral sensitization. Male and female rats were acclimated to the testing apparatus 24 h prior to testing. Following baseline measurements, rats received intraplantar injections of *E. bicolor* latex extract (25, 50, 100, 300, or 500 µg/ml in 100 µl 0.9% sterile saline and 1.2% methanol; n= 5–6 per treatment/sex) or vehicle (100 µl 0.9% sterile saline and 1.2% methanol; n= 5–6/sex) into the hindpaw. Mechanical sensitivity was re-examined at 20, 40, and 60 min post-injection.

To test whether *E. bicolor* latex extract evoked analgesia, basal mechanical sensitivity was recorded followed by one intraplantar CFA injection (see above) into the right hindpaw. Twenty-four hours later, post-CFA mechanical allodynia was confirmed followed by an intraplantar injection into the inflamed hindpaw of either *E. bicolor* latex extract (300 μg/ml in 100 μl 0.9% sterile saline and 1.2% methanol; n = 6 males, n = 6 females) or vehicle (100 μl 0.9% sterile saline and 1.2% methanol; n = 6 males, n = 6 females). Mechanical allodynia was then reassessed at 6, 24, 48, and 72 h post-latex injection followed by every week for 4 weeks.

### Primary Neuronal Cultures

Male rats were rapidly decapitated under brief isoflurane anesthesia and trigeminal ganglia (TG) were bilaterally removed. Primary neuronal cultures were prepared by the method of Patwardhan et al., 2005 (Patwardhan et al., 2005). Briefly, the extracted TGs were suspended in Hanks buffered-saline solution (HBSS) buffer (Invitrogen, San Diego, CA, USA), disassociated and resuspended in Dulbecco’s modified Eagle’s medium containing penicillin–streptomycin, glutamine, 10% fetal bovine serum, nerve growth factor (5 µl of 100 ng/ml; Harlan, Indianapolis, IN, USA), and treated with the mitotic inhibitors 5-fluoro-2-deoxyuridine (3 µg/ml; Invitrogen) and uridine (7 µg/ml; Sigma–Aldrich). Cells were directly applied to 24-well poly-D-lysine-coated plates (n = 3–4 rats or 6–8 TGs/plate; BD Biosciences, Bedford, MA, USA) and maintained in an incubator at 37°C and 5% CO_2_. Twenty-four hours later, the media was replaced with 300 µl of fresh NGF-containing media. This process was continued on every other day for 7 d. All experiments were conducted in duplicate.

### CGRP Release Assay and ELISA

Primary neuronal cultures were incubated in HBSS at 37°C for 15 min. After 15 min, the superfusate was discarded and the cells were incubated again in HBSS at 37°C for 15 min. Superfusate was collected for later quantification of basal CGRP release and the same cells were incubated with varying concentrations of *E. bicolor* latex extract (12.5, 25, 50, 100, and 300 µg/ml) or HBSS vehicle (0 µg/ml) at 37°C for 15 min. The superfusate was again collected for later quantification of extract-evoked CGRP release and the same cells were stimulated with 50 nM of capsaicin along with latex extract at 37°C for 15 min. The superfusate was collected for later quantification of the effects of extract on capsaicin-evoked CGRP release.

A separate set of cultures were incubated in HBSS at 37°C for 15 min. After 15 min, the superfusate was discarded and the cells were incubated again in HBSS at 37°C for 15 min. Superfusate was collected for later quantification of basal CGRP release and the same cells were then incubated for 15 min in either CZP (10 µM in HBSS and <0.05% DMSO), I-RTX (0.02 µM in HBSS and <0.05% DMSO), or vehicle (HBSS and <0.05% DMSO). The same cells were then incubated with *E. bicolor* latex extract (100 µg/ml in HBSS and 1.2% methanol) in the continued presence of either CZP, I-RTX, or HBSS at 37°C for 15 min. The superfusate was collected for later quantification of the effects of the pre-treatments on extract-evoked CGRP release and the same cells were then stimulated with 50 nM of capsaicin along with latex extract at 37°C for 15 min. The superfusate was collected for later quantification of the effects of pretreatment and extract on capsaicin-evoked CGRP release. All collected fractions were immediately stored at −80°C following each individual collection throughout the experiments. Each fraction was analyzed for CGRP levels using a rat-specific CGRP enzyme-linked immunoassay (Cayman Chemicals, Ann Arbor, MI) according to the manufacturer’s protocol.

### Ultra-Performance Liquid Chromatography Electrospray Ionization Tandem Mass Spectrometry (UPLC-ESI-MS/MS)

The chromatographic separation and compound confirmation were carried out by using ultra performance liquid chromatography electrospray ionization tandem mass spectrometry (UPLC-ESI-MS/MS) in a positive ionization mode. A Waters Acquity UPLC (Waters Corporation, MA, USA) chromatography system, coupled with ESI Xevo TQD triple quadrupole mass spectrometer, was used. The UPLC system was equipped with a binary pump, degasser, autosampler, thermostatically controlled column compartment, and control module. Chromatographic separations of analytes were carried out on a Restek Raptor biphenyl (100 mm length x 2.1 mm diameter x 1.8 mm particle size) column using a gradient mobile phase consisting of 0.1% formic acid in 10 mM ammonium formate and 0.1% formic acid in acetonitrile under linear gradient conditions (A:B % v/v, 0–0.5 min: 80:20; 0.5–14 min: 30:70; 14–15 min: 80:20) at 0.6 ml/min flow rate. The column was maintained at 50°C. The source dependent parameters maintained for the analytes were set as follows: cone gas flow of 10 L/h, desolvation gas flow of 1,000 L/h, capillary voltage of 0.70 kV, source temperature of 150°C, and desolvation temperature of 450°C. Detection of the compounds was performed in the multiple-reaction monitoring (MRM) mode by monitoring the pertinent transition pairs (see **Table 1** for specific compound tuning parameters). Unit mass resolution was employed, and the dwell time was optimized automatically *via* Mass Lynx software (autodwell function) at 0.01–0.163 s. Mass Lynx and Target Lynx software (version 4.1) were used to control all parameters of UPLC and ESI-MS/MS operation, and for compound data analysis. Stock solutions of standard compounds were prepared in methanol. The concentrations of the identified phytochemicals were determined with the above software, utilizing a three-point, external calibration method.

**Table 1:** Phytochemical analysis of *E. bicolor* latex extract by UPLC-ESI-MS/MS (alphabetical order by phytochemical names).

Retention time (RT)	Molecular formula	Parent molecule (m/z)	MS/MS ion fragments (quantitative*, qualitative)	Cone voltage (V)	Collision energy (eV)	Phytochemicals	Classification

9.9	CH3COOH	303.23	93.1	24	30	Abietic Acid	Diterpene
		303.23	**123.12**	24	14		
5.55	C16H12O5	284.98	**114.96**	54	62	Biochanin A	Isoflavone
		284.98	213.02	54	40		
7.15	C15H12O	209.1	103.05	26	26	Chalcone	Flavonoid
		209.1	**131.06**	26	16		
3	C15H8O5	269.06	**197.07**	54	26	Coumestrol	Coumestan
		269.06	213.06	54	26		
1.98	C15H10O4	255.1	**91.08**	52	36	Daidzein	Isoflavone
		255.1	137.02	52	26		
2.94	C15H10O5	271.02	91.02	18	42	Genistein	Isoflavone
		271.02	148.97	18	22		
2.97	C15H10O6	287.07	**69.06**	53	44	Kaempferol	Flavonol
		287.07	**153.07**	53	33		
2.94	C15H12O5	273.1	147.03	36	20	Naringenin	Flavanone
		273.1	153.07	36	22		
2.15	C15H10O7	303.08	**69.06**	50	46	Quercetin	Flavonol
		303.08	153.01	50	31		
0.75	C37H40O9	629.42	293.18	30	20	Resiniferatoxin	Diterpene
		629.42	**311.19**	30	17		
10.32	C27H30O16	611.23	**303.07**	22	21	Rutin	Flavonoid
		611.23	465.17	22	13		

*Quantitative ion in bold text.

## Statistical Analysis

All data were analyzed using GraphPad Prism software version 7 (GraphPad, San Diego, CA, USA). Behavioral data were presented as mean ± SEM paw withdrawal latency or force in grams and analyzed by two-way repeated measures analysis of variance (ANOVA). ELISA data is presented as mean ± SEM of percent basal levels and analyzed by unpaired t test or one-way ANOVA. Bonferroni *post-hoc* analysis was conducted, and the statistical significance was tested at p ≤ 0.05. Significant outliers were identified for exclusion with the Grubb’s test (GraphPad Quick Calcs Online, the extreme studentized deviate method; [(mean-value)/standard deviation]) to detect an outlier over 2 standard deviations from the mean.

## Results

### *E. bicolor* Latex Extract Induced Transient Pain Behaviors in Both Male and Female Rats

*E. bicolor* latex extract evoked significant thermal hyperalgesia in both male [F (5,26) = 37.36; p ≤ 0.05] (**Figure 1A** ) and female rats [F (5,26) = 7.53; p ≤ 0.05] (**Figure 1B** ). At 20 min post-extract injection in males, the PWLs following injection of the concentrations over 50 µg/ml were significantly lower than vehicle. At 2 h, only the 300 and 500 µg/ml concentrations of extract continued to induce significant hyperalgesia. Hyperalgesia was resolved by 4 h post-extract injection. In females, only the 300 and 500 µg/ml concentrations of extract from 20–60 min induced significant hyperalgesia. Hindpaw injection of *E. bicolor* latex extract also evoked significant mechanical allodynia in both male [F(5,24) = 28.82; p ≤ 0.05] (**Figure 2A** ) and female rats [F(5,26) = 12.07; p ≤ 0.05] (**Figure 2B** ). At the 20, 40, and 60 min time points, the 50, 100, 300, and 500 µg/ml concentrations evoked significantly greater allodynia than vehicle controls in both males and females, but the two highest doses remained significant at 60 min post-injection in females only. The 25 µg/mL concentration of the latex extract did not evoke either of the pain behaviors tested in either sex (p > 0.05).

**Figure 1:** *E. bicolor* latex extract induced thermal hyperalgesia in male and female rats. Thermal hyperalgesia in male (n = 5–6) **(A)** and female (n = 5–6) **(B)** rats injected with various concentrations of *E. bicolor* latex extract in the right hindpaw compared to vehicle injections. * indicate p ≤ 0.05 compared to vehicle by RM two-way ANOVA with Bonferroni *post hoc* analysis.

**Figure 2:** *E. bicolor* latex extract induced mechanical allodynia in male and female rats. Mechanical allodynia in male (n = 5–6) **(A)** and female (n = 5–6) **(B)** rats injected with *E. bicolor* latex extract in the right hindpaw compared to vehicle injections. * indicate p ≤ 0.05 compared to vehicle by RM two-way ANOVA with Bonferroni *post hoc* analysis.

### *E. bicolor* Latex Extract Elicits Long-Lasting Peripheral Analgesia in Male and Female Rats

CFA evoked significant thermal hyperalgesia at 24 h post-hindpaw injection that lasted up to four weeks in males [F(11,121) = 45.6; p ≤ 0.05] and three weeks in females [F(11,165) = 46.0; p ≤ 0.05]. Peripheral injection of *E. bicolor* latex extract into the inflamed hindpaw induced significant analgesia in males observed as an increase in paw withdrawal latencies compared to vehicle controls [F (1, 11) = 75.0; p ≤ 0.05] (**Figure 3A** ). The onset of significant analgesia occurred at 6 h post-latex injection and lasted through 4 weeks (p ≤ 0.05) in male rats, whereas, in female rats [F (1, 15) = 7.9; p ≤ 0.05] (**Figure 3B** ), the onset of significant analgesia occurred at 72 h and lasted through recovery of CFA-evoked inflammatory pain at 3 weeks (p ≤ 0.05). There was also a significant effect of vehicle treatment at 1 h following latex extract injection with the vehicle treatment group displaying consistent and significantly greater hyperalgesia than the extract treatment group. We also observed a significant reduction in mechanical allodynia at 24 h in male rats [F (1, 10) = 244.4; p ≤ 0.05] (**Figure 3C** ) and 72 h in female rats [F (1, 10) = 403.1; p ≤ 0.05] (**Figure 3D** ) that returned to baseline by 4 weeks.

**Figure 3:** *E. bicolor* latex extract elicited long-lasting peripheral analgesia in male and female rats. Peripheral analgesia on thermal hyperalgesia in a rat model of inflammatory pain was detected in males at 6 h post-*E. bicolor* latex extract injection (n = 7) and still significantly present at 4 weeks as compared to vehicle treated (n = 6) **(A)**. In females, peripheral analgesia was detected at 72 h post-*E. bicolor* latex extract injections (n = 9) as compared to vehicle treated (n = 9) **(B)**. Peripheral analgesia on mechanical allodynia was detected in males at 24 h post-*E. bicolor* latex extract injection (n = 6) and was comparable to vehicle treated (n = 6) by 4 weeks post-injection **(C)**. In females, peripheral analgesia was again detected at 72 h post-*E. bicolor* latex extract injections (n = 6) as compared to vehicle treated (n = 6) **(D)**. * indicate p ≤ 0.05 compared to vehicle by RM two-way ANOVA with Bonferroni *post hoc* analysis. + indicates p ≤ 0.05 compared to pre-CFA baseline by RM two-way ANOVA with Bonferroni *post hoc* analysis.

### *E. bicolor* Latex Extract Does Not Elicit Peripheral Analgesia *via* Opioid Receptors

To test whether phytochemicals present in the *E. bicolor* latex extract induce peripheral analgesia through opioid receptors, male rats were pretreated systemically with the broad-spectrum opioid antagonist naloxone prior to the latex extract injection and CFA-evoked thermal hyperalgesia was assessed. In both groups, *E. bicolor latex* extract evoked significant analgesia [F(4,40) = 154.5; p ≤ 0.05] at 6 h and 24 h post-extract injection (p ≤ 0.05) (**Figure 4A** ). There was no significant effect of naloxone compared to vehicle pretreatment on *E. bicolor*-evoked analgesia [F(1,10) = 0.002; p > 0.05].

**Figure 4:** *E. bicolor* latex extract elicited non-opioid analgesia *via* TRPV1, but not hyperalgesia. Extract-evoked analgesia was not blocked in males following systematic pre-treatment with the opioid antagonist naloxone as illustrated by the presence of significant analgesia in the extract- (n = 6) and vehicle-treated groups (n = 6) at 6 h and 24 h as compared to the 1 h timepoint **(A)**. Extract-evoked thermal hyperalgesia was not blocked in males following local pre-treatment with the TRPV1 antagonist capsazepine (CZP) as illustrated by the presence of significant thermal hyperalgesia in the extract-treated group (n = 7) compared to the vehicle-treated group (n=7) **(B)**. In both males **(C)** and females **(D)**, CZP pre-treatment (n = 7 males; n = 6 females) significantly blocked the onset of extract-evoked analgesia as compared to vehicle-treated (n=7 males; n=6 females). In both males **(E)** and females **(F)**, 5’-Iodoresiniferatoxin (I-RTX) pre-treatment (n = 6 / sex) also significantly blocked the onset of extract-evoked analgesia as compared to vehicle-treated (n = 6 / sex). * indicate p ≤ 0.05 compared to vehicle by RM two-way ANOVA with Bonferroni *post hoc* analysis. + indicates p≤0.05 compared to 24 h post-CFA by RM two-way ANOVA with Bonferroni *post hoc* analysis.

### Blocking TRPV1 Attenuated *E. bicolor* Latex Extract-Induced Analgesia, but Not Hyperalgesia

To test whether *E. bicolor* latex extract phytochemicals target TRPV1 with a similar mechanism to RTX isolated from *E. resinifera*, rats were pretreated with the TRPV1 antagonist CZP prior to peripheral latex extract injection and the role of TRPV1 in both *E. bicolor* extract-evoked thermal hyperalgesia and *E. bicolor* extract-evoked analgesia were tested. CZP did not alter *E. bicolor* extract-evoked hyperalgesia as a significant drop in paw withdrawal latency following *E. bicolor* extract was still observed [F (1, 12) = 453.2; p ≤ 0.05] (**Figure 4B** ). There was no significant difference between the vehicle and CZP groups at baseline or 20 min following extract injections (p > 0.05). CZP did attenuate *E. bicolor* extract-evoked analgesia in both male and female rats. In male rats, blocking TRPV1 with CZP prior to extract injections attenuated analgesia observed as a significantly lower paw withdrawal latency compared to vehicle pretreatment at 6 h and 24 h post-extract injection [F (1, 10) = 10.9; p ≤ 0.05] (**Figure 4C** ). At 6- and 24-h post-extract injection, the vehicle pretreatment groups displayed significant analgesia compared to the post-CFA timepoint (p ≤ 0.05), while the CZP pretreatment group did not show significant difference from the post-CFA timepoint (p> 0.05). For female rats, blocking TRPV1 with CZP prior to extract injections attenuated analgesia observed as a significantly lower paw withdrawal latency compared to vehicle pretreatment at 72 h post-extract injection [F (1, 40) = 1.711; p ≤ 0.05] (**Figure 4D** ). In support, blocking TRPV1 with another TRPV1 antagonist I-RTX also significantly attenuated extract-evoked analgesia in both males [F (1, 10) = 150.9; p ≤ 0.05] (**Figure 4E** ) and females [F (1, 10) = 6.17; p ≤ 0.05] (**Figure 4F** ) at the same time points.

### *E. bicolor* Latex Extract Treatment Evokes CGRP Release and Attenuates Capsaicin-Evoked CGRP Release *via* TRPV1 *in Vitro*

To test the direct effects of *E. bicolor* latex extract on sensory neurons *in vitro*, primary neuronal cultures of trigeminal sensory neurons were treated with varying concentrations of *E. bicolor* latex extract and CGRP was quantified as a functional measure of peptidergic neuronal activity. *E. bicolor* latex extract treatment evoked a significant increase in the release of CGRP from cultured sensory neurons at all concentrations compared to vehicle treated controls [F (5, 59) = 3.5; p ≤ 0.05] (**Figures 5A, B** ). Capsaicin stimulation of the same cultured cells resulted in a significant increase in CGRP release [t = 4.371 df = 26] (**Figures 5C, D** ). *E. bicolor* latex extract significantly reduced capsaicin-evoked CGRP release at the 50 and 100 µg/ml concentrations [F (5, 66) = 2.7; p ≤ 0.05] (**Figure 5D** ). Prior to conducting the TRPV1 antagonist studies, neuron density per well was increased (from 6 to 8 TGs per plate) to optimize CGRP detection levels for pharmacological manipulations. As the density of neurons is different between the cell cultures in **Figures 5** and **6** and thus the y axes are not similar, we only conducted statistical analysis on the percentage of basal release rather than the actual fmol/ml to control for differences in CGRP release that due to unequal neuron density. When TRPV1 was blocked with CZP prior to and during treatment with *E. bicolor* latex extract, *E. bicolor* latex extract-evoked CGRP release from sensory neurons was significantly attenuated [t = 2.178 df = 22] (**Figures 6A, B** ). Also, TRPV1 antagonism significantly attenuated capsaicin-evoked CGRP release and the effects of the extract on capsaicin-induced CGRP release [F (2, 33) = 5.975; p ≤ 0.05] (**Figures 6C, D** ). In support, pretreatment with the TRPV1 antagonist I-RTX also significantly attenuated both extract-evoked CGRP release [t = 43.49 df = 22] (**Figures 7A, B** ) and the effects of extract on capsaicin-induced CGRP release [F (2, 33) = 1666; p ≤ 0.05] (**Figures 7C, D** ).

**Figure 5:** *E. bicolor* latex extract treatment evoked CGRP release and attenuated capsaicin-evoked CGRP release. *E. bicolor* latex extract induced significant CGRP release from sensory neurons treated with 12.5, 25, 50, 100, and 300 µg/ml extract (shaded bars) compared to vehicle treated (open bars) (**A** in fmol, **B** in percent of basal release). *E. bicolor* latex extract also significantly reduced capsaicin-induced release of CGRP at 50 and 100 µg/ml extract (shaded bars) (**C** in fmol, **D** in percent of basal release). * indicate p ≤ 0.05 compared to vehicle by one-way ANOVA with Bonferroni *post hoc* analysis. Statistical analyses were performed only on percent of basal of release.

**Figure 6:** *E. bicolor* latex extract treatment modulated CGRP release and capsaicin-evoked CGRP release *via* TRPV1 *in vitro*. Treatment with the TRPV1 antagonist capsazepine (CZP) significantly reduced the extract-evoked CGRP release from cultured sensory neurons (black bar) as compared to treatment with the vehicle (white bar) (**A** in fmol, **B** in percent of basal release). Treatment with CZP prior to and during treatment with both *E. bicolor* and capsaicin (black bar) or capsaicin only (grey bar) significantly reduced CGRP release compared to vehicle pre-treatment (white bar) (**C** in fmol, **D** in percent of basal release). * indicate p ≤ 0.05 compared to vehicle by Student *t*-test or one-way ANOVA with Bonferroni *post hoc* analysis. Statistical analyses were performed only on percent of basal of release.

**Figure 7:** *E. bicolor* extract treatment-evoked effects on CGRP were attenuated by a TRPV1 antagonist. Treatment with the TRPV1 antagonist 5’-Iodoresiniferatoxin (I-RTX) significantly reduced the extract-evoked CGRP release from cultured sensory neurons (black bar) as compared to treatment with the vehicle (white bar) (**A** in fmol, **B** in percent of basal release). Treatment with the I-RTX prior to and during treatment with both *E. bicolor* and capsaicin (black bar) or capsaicin only (grey bar) significantly reduced CGRP release compared to vehicle pre-treatment (white bar) (**C** in fmol, **D** in percent of basal release). * indicate p ≤ 0.05 compared to vehicle by Student *t*-test or one-way ANOVA with Bonferroni *post hoc* analysis. # indicates p ≤ 0.05 in between I-RTX+capsaicin and I-RTX+extract+capsaicin by one-way ANOVA with Bonferroni *post hoc* analysis. Statistical analyses were performed only on percent of basal of release.

### Chemical Composition of *E. bicolor* Latex Extract Identified by UPLC-ESI-MS/MS

UPLC-ESI-MS/MS identified eleven compounds based on standard compounds (**Figure 8** and **Table 1**) that belong to four major groups of phytochemicals: coumestans, diterpenes, flavonoids, and isoflavones. Coumestrol (coumestans), abietic acid and resiniferatoxin (diterpenes), chalcone, kaempferol, naringenin, quercetin, and rutin (flavonoids) and biochanin A, daidzein, and genistein (isoflavones) were the eleven compounds identified. The concentration of the identified phytochemicals quantified by the MassLynx ™ MS software ranked as follows: biochanin A > coumestrol > naringenin > chalcone > quercetin > kaempferol > RTX > rutin > abietic acid > genistein > daidzein.

**Figure 8:** Chemical composition of *E. bicolor* latex extract identified by UPLC-ESI-MS/MS. Representative ion chromatograms and the corresponding structures of the phytochemicals identified in the crude extract by UPLC-ESI-MS/MS. Daidzein **(A)**, genistein **(B)**, abietic acid **(C)**, rutin **(D)**, resiniferatoxin **(E)**, kaempferol **(F)**, quercetin **(G)**, chalcone **(H)**, naringenin **(I)**, coumesterol **(J)**, biochanin A **(K)**.

## Discussion

A number of studies have reported the analgesic and anti-inflammatory properties of different *Euphorbia* species (Prabha et al., 2008; Gaur et al., 2009; Upadhyay et al., 2014; Majid et al., 2015; Palit et al., 2018; Sdayria et al., 2018). However, no studies have reported the analgesic properties and phytochemical analysis of *E. bicolor* latex extract. We hypothesized that the *E. bicolor* latex extract contains phytochemicals that induce long-lasting, non-opioid, peripheral analgesia in a rat model of inflammatory pain. Here, we report several novel findings supporting our hypothesis: (1) *E. bicolor* latex extract induced transient pain behaviors in male and female rats; (2) latex extract evoked non-opioid long-lasting analgesia partly *via* TRPV1 in male and female rats; (3) latex extract evoked a transient increase in CGRP release but attenuated capsaicin-evoked CGRP release in cultured sensory neurons; and (4) phytochemical analysis of latex extract revealed the presence of bioactive compounds.

In the present study, intraplantar injections of *E. bicolor* latex extract significantly induced pain behaviors manifested as thermal hyperalgesia and mechanical allodynia. The results from the current study is in accordance with those of a previous study in which the intradermal injection of capsaicin into the plantar skin of the hindpaw in mice led to the development of thermal and mechanical hyperalgesia (Caterina et al., 1997). It is widely agreed that primary mechanical and thermal hyperalgesia are a consequence of the sensitization of primary sensory neurons (Treede et al., 1992). *E. bicolor* latex extract also significantly enhanced the release of the pro-inflammatory peptide CGRP. Together, these data indicate that *E. bicolor* latex extract is an irritant that evokes significant pain behaviors and pronociceptive signaling in sensory neurons. However, we found that antagonizing TRPV1 did not block the onset of hyperalgesia. It is possible that extract-induced hyperalgesia is occurring *via* TRPV1, but the presence of one or several other irritant phytochemicals in the extract may also trigger hyperalgesia.

Resiniferatoxin, a potent analogue of capsaicin, has been reported to reverse thermal hyperalgesia and mechanical allodynia in rats following full thickness thermal injury (Salas et al., 2017). In CFA-inflamed rats, one peripheral injection of *E. bicolor* latex extract (300 µg/ml) significantly induced analgesia in male rats starting at 6 h that lasted up to recovery at 4 weeks. In female rats, analgesia started at 72 h and lasted up to 3 weeks. Injection of CFA in rats results in inflammation and thermal hyperalgesia and mechanical allodynia within 12 h that lasts to approximately between 2–3 weeks (Stein et al., 1988; Lyness et al., 1989; Cobos et al., 2012; Parvathy and Masocha, 2013). While a limitation of this study is that a direct comparison to RTX-evoked analgesia was not included, long-lasting analgesia following a single injection of *E. bicolor* latex extract was similar to that of RTX, which significantly reduced thermal hyperalgesia in a rat model of burn pain within 2.5 h of injection and lasted through recovery at three weeks postinjury (Salas et al., 2017). Our data supports the necessity of further studies directly comparing the potency and efficacy of identified novel candidate phytochemicals in *E. bicolor* latex in comparison to TRPV1 therapeutics currently being explored in clinical trials. Of note, TRPV1 agonists that trigger hyperalgesia and desensitization of the ion channel to induce analgesia may require the use of either local or general anesthetics at the onset of treatment in the clinic (Iadarola and Mannes, 2011).

An unexpected finding of this study was that female rats displayed a later onset of analgesia compared to males. This discrepancy could be attributed to the different phases of estrous cycle in female rats (Loyd and Murphy, 2009), however studies with other plant extracts have not revealed an effect of estrous cycle on analgesia (Ratnasooriya et al., 2002; Dharmasiri et al., 2003). A possible explanation could be that the major female gonadal hormone estrogen is altering *E. bicolor*-evoked analgesia *via* a neuroprotective mechanism (Brann et al., 2007; Tiwari-Woodruff and Voskuhl, 2009; Nobakhti-Afshar et al., 2016). In support, 17β-estradiol can slow the progression of injury *via* suppressing the apoptotic pathway, enhancing the expression of cell survival genes (Wise et al., 2005), as well as offering protection against oxidative stress, glucose deprivation, and neurodegeneration (Goodman et al., 1996; Patrone et al., 1999; Blacklock et al., 2005; Fan et al., 2007). In the present study, it is possible that estradiol provided some level of protection from *E. bicolor* extract induced nerve ablation in female rats which resulted in the delayed onset of analgesia. Future studies are warranted to investigate this possibility.

Opioid receptors are widely distributed in both the central and peripheral nervous system, (Zöllner and Stein, 2007) which can be targeted for peripheral analgesia (Stein et al., 2009). In the present study, antagonizing mu, delta, and kappa opioid receptors did not block the onset of analgesia, indicating that the *E. bicolor* latex extract induces non-opioid analgesia. On the other hand, blocking the TRPV1 ion channel with either capsazepine or 5’-Iodoresiniferatoxin attenuated extract-induced analgesia in both male and female rats, indicating that the latex extract induces analgesia in part *via* TRPV1. We did not observe an analgesic effect of capsazepine at this concentration (10 µM), similar to a previous study (Menéndez et al., 2006). Capsazepine’s binding affinity for TRPV1 is reported at 1.3 −4.3 µM (Seabrook et al., 2002; Wang et al., 2002). However, capsazepine has also been reported to have affinity for voltage-gated calcium channels and acetylcholine receptors at concentrations over 10 µM (Docherty et al., 1997; Liu and Simon, 1997). As it remains possible that our analgesic effects may be occurring through other calcium channels or acetylcholine receptors, we repeated the experiments with another TRPV1 antagonist, 5’-Iodoresiniferatoxin (IC_50_ = 0.7 nM), which has 800-fold higher affinity for rat TRPV1 compared to capsazepine (IC_50_ = 562 nM) (Seabrook et al., 2002). 5’-Iodoresiniferatoxin’s binding affinity for TRPV1 is reported at 0.39 nM (Seabrook et al., 2002). The results from both sets of TRPV1 antagonist studies revealed that TRPV1 antagonism attenuated the onset of *E. bicolor*-evoked analgesia. One caveat to this, 5’-Iodoresiniferatoxin has been reported to also display TRPV1 agonistic characteristics (Petho et al., 2004) at 0.06–9.9 µM (Shimizu et al., 2005). The present study used 0.02 µM so it is not likely that agonistic characteristics are active in this study, but if TRPV1 agonism were occurring then the data could be interpreted as a dampened but still significant analgesic effect.

Our *in vitro* data also support *E. bicolor* latex-evoked hyperalgesia followed by the development of analgesia. Capsaicin significantly evoked CGRP release similar to our previous report (Loyd et al., 2012) and the latex significantly reduced capsaicin-evoked CGRP release. Further, blocking the TRPV1 ion channel with either capsazepine or 5’-Iodoresiniferatoxin significantly reduced both capsaicin-evoked and *E. bicolor* latex-evoked CGRP release. While capsaicin and *E. bicolor* latex extract treatment each independently increased CGRP release, given together they evoked a comparable rather than further enhanced degree of CGRP release. As we confirmed a significant effect of capsaicin on these cells in the positive control group, the lack of further enhancement may indicate that desensitization of the TRPV1 ion channel is occurring as the cells were first treated for 15 min in *E. bicolor* followed by a further 15 min treatment in *E. bicolor* (30 min total) plus capsaicin. It can also be noted that there was a greater magnitude of change in evoked CGRP release in **Figures 6** and **7** compared to **Figure 5**. This is likely due to an increase in neuron density and stability per well as well as an increase in length of treatment per the methodology change between the experiments. This illustrates the importance of examining the data as percentage of baseline per well to control for differences between experimental designs. Overall, our *in vivo* and *in vitro* data together suggest that *E. bicolor* latex extract induces analgesia by reducing nociceptive signaling at least in part *via* TRPV1.

The *Euphorbia* plant family contains several plants that are known for their medicinal properties and our data indicate that *E. bicolor* is one of them. In the present study, we have identified eleven compounds belonging to three major groups of phytochemicals, coumestans, diterpenes, flavonoids (with flavonol and flavanone groups). Each group contains phytochemicals with activities that could contribute to analgesia. Coumestrol (coumestans) derived from the roots of *Pueraria lobata*, has anti-inflammatory and antioxidant properties (Jin et al., 2012), suppresses the lipopolysaccharide-induced activation of microglia (Jantaratnotai et al., 2013), and can downregulate the interleukin 1β-induced upregulation of pro-inflammatory cytokines (You et al., 2017). Oral or topical application of abietic acid (diterpene) significantly reduces edema and inflammatory mediators in a rat model of inflammatory pain (Fernandez et al., 2001). Recent reports provide evidence that reactive oxygen species can increase pain processing *via* TRPV1 (Yoshida et al., 2006; Ibi et al., 2008). It is likely that *E. bicolor* latex extract is reducing inflammatory mediators and oxidative stress, based on data from other *Euphorbia* species (Upadhyay et al., 2014; Majid et al., 2015; Palit et al., 2018; Sdayria et al., 2018) as a mechanism underlying the analgesia observed in the present study. This hypothesis is currently under investigation.

RTX (diterpene) has been the research subject of a rich literature of analgesia studies (Brown et al., 2005; Neubert et al., 2008; Iadarola and Mannes, 2011; Salas et al., 2017) and is currently in clinical trials to treat pain in terminal cancer patients (NCT00804154 and NCT02522611). Dimeric chalcone, isolated from *Myracrodruon urundeuva allemão*, exhibits central and peripheral analgesic properties and anti-inflammatory activities (Viana et al., 2003). Quercetin has anti-inflammatory activities *via* reduction of oxidative stress and cytokine production (Valerio et al., 2009) and kaempferol also has anti-inflammatory and antinociceptive properties (De Melo et al., 2009). Rutin attenuates chemotherapy-induced neuropathy (Azevedo et al., 2013) and naringenin reduced inflammatory pain in rats (Pinho-Ribeiro et al., 2016; Manchope et al., 2017). Biochanin A, genistein, and daidzein (isoflavones) attenuate neuropathic pain in diabetic rats (Chundi et al., 2016) and in rats with partial sciatic nerve ligation (Shir et al., 1998). Taken together, these data suggest that the identified phytochemicals contributed to an additive effect on *E. bicolor* latex extract-induced analgesia.

## Conclusions

To our knowledge, this is the first report on the phytochemical analysis and biological activities of *E. bicolor* latex extract. Our results indicate that *E. bicolor* latex extract induces long-lasting, non-opioid, peripheral analgesia in part *via* TRPV1 in both male and female rats, thus adding new data to the literature on the analgesic activities of the *Euphorbia* species. The identified secondary metabolites with anti-inflammatory and antinociceptive properties are likely contributing, possible in a synergistic manner, to the observed analgesic properties of the latex extract. Many other phytochemicals in the *E. bicolor* latex extract are yet to be identified and future studies will individually examine these bioactive components to support discovery of novel phytomedicines. The identification of novel phytochemicals that target non-opioid mechanisms and act at the peripheral nervous system has the potential to improve pain management by reducing reliance on opioids and reducing the negative side effects elicited *via* the central nervous system.

## Data Availability

The datasets generated for this study are available on request to the corresponding author.

## Ethics Statement

All studies were conducted under the approval of the Texas Woman’s University Institutional Animal Care & Use Committee and under the strict guidelines of Animal Welfare Act, implementing Animal Welfare Regulations, and the principles of the Guide for the Care and Use of Laboratory Animals. The study also followed the guidelines of the Committee for Research and Ethical Issues of the International Association for the Study of Pain. For all behavior testing, experimenters were blind to the treatment groups during testing.

## Author Contributions

PB contributed to study design, performed experiments, analyzed and interpreted data, and prepared manuscript. ST and TH contributed to study design, performed behaviour experiments, analyzed and interpreted data, and approved the final manuscript. AR, JG, and JW performed the phytochemical analysis, prepared chromatographs, contributed sections to the manuscript, and approved the final manuscript. CM contributed to study design, analyzed and interpreted data, and prepared the manuscript. DA contributed to study design, performed experiments, analyzed and interpreted data, and prepared manuscript.

## Funding

This research was supported by Texas Woman’s University (TWU) Research Enhancement Grants awarded to CM and DA, a TWU Chancellor’s Research Fellowship awarded to DA, TWU Quality Enhancement Program Learn by Doing grants awarded to PB and ST, and a TWU Center for Student Research Small Grant awarded to DLA and PB.

## Conflict of Interest Statement

AR, JG, and JW were employed by the American Institute of Toxicology (AIT) Laboratories, A HealthTrackRx Company.

The remaining authors declare that the research was conducted in the absence of any commercial or financial relationships that could be construed as a potential conflict of interest.
